# Effect of Acupotomy Combined with Electroacupuncture Therapy on Finger Mobility and Pain Relief in Patients with Carpal Tunnel Syndrome

**DOI:** 10.1155/2022/2550875

**Published:** 2022-07-14

**Authors:** Jianfei Li, Yinqiao Kou, Suzhao Zhang, Kaibing Wang

**Affiliations:** Department of Acupuncture and Moxibustion Rehabilitation, Hebei Provincial Hospital of Traditional Chinese Medicine, Shijiazhuang, 050011 Hebei, China

## Abstract

**Objective:**

To explore the effect of acupotomy in combination with electroacupuncture therapy on the finger mobility and pain relief in patients who had carpal tunnel syndrome (CTS).

**Methods:**

The clinical data of 60 CTS patients in our hospital from November 2020 to November 2021 received retrospective analysis. With 30 cases in each group, they were randomly divided into the treatment group and the control group. The control group underwent hot compress, oral medication, and local injection during hospitalization, while the treatment group received acupotomy and electroacupuncture therapy on top of the above treatments, and the clinical effects, finger mobility, and pain relief were compared between both groups.

**Results:**

The clinical indexes in the treatment group after treatment were remarkably better than those in the control group (*P* < 0.05), with the remarkably higher number of cured cases in the treatment group (*P* < 0.05). After treatment, the treatment group had remarkably higher mean total active motion (TAM) and score of the 36-item short form (SF-36) health survey and a remarkably lower mean score of visual analog scale (VAS) than those in the control group (*P* < 0.001).

**Conclusion:**

The quality of life and finger mobility of CTS sufferers can be improved with acupotomy in conjunction with electroacupuncture therapy. In-depth research will help build better procedures for these patients because this approach lessens the discomfort and shortens the symptom duration in CTS sufferers.

## 1. Introduction

Carpal tunnel syndrome (CTS) is a peripheral nerve entrapment disease in the upper extremity that occurs when median nerve is injured and compressed in the narrow space of carpal tunnel [1], which is most often diagnosed in women and has a growing trend in prevalence rate in recent years. CTS patients show abnormal sensations in the hands and wrists, the typical symptoms of pain, numbness and abnormal sensation in the radial three fingers, and muscle weakness in severe cases which results in a series of syndromes such as motor dysfunction, bringing about serious psychological burden to patients and declining the quality of life [2, 3]. Clinically preferable treatments for mild to moderate CTS include wrist splinting, therapeutic ultrasonography, and oral medicines. However, these treatments have short-term sustained efficacy and patients are susceptible to recurrence [4]. Surgical treatments have some efficacy but also bring about complications such as postoperative pain and weakness. As a result, safe and effective nonsurgical methods have great implications for the treatment of CTS [5].

Acupotomy is a modern treatment technique developed with the advancement of medical technology, which combines the features of the acupuncture needle from traditional Chinese medicine and the scalpel from Western medicine in order to better relieve the pathological state of the tissues and restore the dynamic balance of the affected areas. A study [6] has found that acupotomy can effectively reduce pain and greatly shorten the treatment time. A study [7] has confirmed that electroacupuncture has obvious advantages in the treatment of CTS. On the one hand, acupuncture can successfully increase blood flow to the wrist of patients and reduce adhesion and inflammatory responses in the surrounding tissues; on the other hand, acupuncture relieves spasm, edema, and discomfort by dredging qi and blood in nearby veins. Current research on acupotomy combined with electroacupuncture as a conservative treatment for CTS is still very limited. Therefore, this study further confirms the effect of combined therapy on the finger mobility and pain relief in CTS patients by a comparative study, aiming to search for more evidence for the treatment of this disease.

The paper's organization paragraph is as follows: the research materials and methods is presented in Section 2.  Section 3 discusses the experiments and results. Finally, in Section 4, the research work is concluded.

## 2. Materials and Methods

In this section, we define the general data, inclusion and exclusion criteria, methods, observational indexes, and statistical disposal in detail.

### 2.1. General Data

60 CTS patients chosen from our hospital from November 2020 to November 2021 received retrospective analysis, which was in line with the Declaration of Helsinki (2013) [8]. With 30 cases in each group, the patients were randomly divided into the treatment group and the control group. There were no remarkable differences in clinical data such as age, course of disease, and previous treatments between the two groups (*P* > 0.05), as shown in Table 1.

### 2.2. Inclusion and Exclusion Criteria

Inclusion criteria are as follows. (1) The patients displayed typical CTS symptoms such as sensory loss and numbness in the area of the median nerve distribution, hypoesthesia, and thenar muscle atrophy that were discovered during physical examinations, as well as positive results from the Phalen or Tinel tests; (2) the patients were aged between 18 and 70, with no gender limitations; and (3) the patients had the median nerve motor latency of ≥4.5 ms and the sensory nerve conduction velocity of <40 m/s by nerve electrophysiological examination.

Exclusion criteria are as follows: (1) patients with cervical spondylotic radiculopathy or polyneuritis; (2) patients with infections, severe cardiovascular and cerebrovascular diseases, or liver and kidney diseases; and (3) patients with other diseases that cannot be treated with acupotomy or electroacupuncture.

### 2.3. Method

The control group underwent hot compress, oral medication, and local injection, with the specific steps as follows. For two weeks, the patients received heat compress therapy on their carpometacarpal side five times each week for 20 minutes each session. Oral mecobalamin (manufacturer: Eisai China Inc.; NMPA Approval No. H20143107; specification: 0.5 mg∗10 tablets∗2 plates/box) was administrated with 0.5 mg each time, with 3 times a day for 2 weeks. The midpoint of the proximal transverse carpal ligament in patients was given local injection of 3 mg of dexamethasone (manufacturer: Guangzhou Baiyunshan Tianxin Pharmaceutical Co., Ltd.; NMPA Approval No. H44022091; specification: 5 mg : 1 ml∗10 piece) and 3 ml of normal saline, once a week for 2 times.

Based on the therapies received by the control group, the treatment group added acupotomy and electroacupuncture, with the specific stages being as follows. The entry point was chosen among the midpoint of the proximal transverse carpal ligament, the flexor carpi radialis muscle tendon, and the palmaris longus tendon, and 0.5 ml of lidocaine (manufacturer: Jinling Pharmaceutical Co., Ltd. Nanjing Jinling Pharmaceutical Factory; NMPA Approval No. H20054551; specification: 5 ml : 40 mg) was used for skin anesthesia. The acupotomy was performed with the blade parallel to the path of the tendon and perpendicular to the wrist before switching to a gradual piercing motion toward the distal limb and fingers. At the same time, the patients were asked how they felt about the acupotomy, adjusting the stabbing direction slightly when obvious pain or sense of electric shock occurred. Looking for the sense of loosening when the acupotomy was walking under the transverse carpal ligament, the treatment was terminated after 2-3 times of loosening. Bandaging was done after removing the acupotomy and pressing the pinhole with a sterile cotton pellet for 30 s, and the patients were told to keep the pinhole dry for 24 h. Daling and Jingqu acupoints on the affected side were located according to the acupuncture methods from traditional Chinese medicine and punctured into 3-cun acupuncture needles which were connected to an electro-acupuncture apparatus (manufacturer: Jinan Qiansi Biotechnology Co., Ltd.; model: G6805-II) for treatment, with 20 min each time, once every other day, and three times a week. The continuous waves and intensity were appropriate for the patients to feel weird but no pain.

### 2.4. Observation Indexes

Clinical indexes are as follows. The time from treatment to pain relief, numbness relief, and the distension sensation scores were recorded for both groups, with the marking criteria as follows. The affected part with obvious distension sensation, tension blisters, and a central height of >1 cm was degree 3 (points); the affected part with increased tension compared to normal skin, clear skin lines, no tension blisters, and a central height of 0.5-1 cm was degree 2 (points); the affected part with mild distension sensation, clear skin lines, and a central height of <0.5 cm was degree 1 (points); skin with no distension sensation, clear lines, and normal elasticity was degree 0 (points).

Evaluation of efficacy is as follows. (1) Cured: after treatment, the clinical symptoms and signs disappeared, and the wrist and fingers moved freely, with negative result of the carpal flexion and extension test or the Tinel test. (2) Improved: when compared to prior therapy, the clinical symptoms and indicators significantly improved. However, the Tinel test or carpal flexion and extension test revealed positive results, and the wrist was weak after effort. (3) Ineffective: there was no improvement in the clinical signs after treatment, with positive result of the carpal flexion and extension test or the Tinel test.

Mobility of fingers is as follows. The total active motion (TAM) of fingers after treatment was evaluated in both groups with reference to the trial criteria for upper limb function assessment of the Hand Surgery Society of Chinese Medical Association [9]. TAM = active flexion [metacarpophalangeal (MP) + proximal interphalangeal (PIP) + distal interphalangeal (DIP)] − extension deficit (MP + PIP + DIP). Joints extended to 0° were straight, excluding the overstretched part.

Relief of pain is as follows. The improvement in pain of patients after treatment was assessed by the visual analog scale (VAS) [10], which needed to prepare a 10 cm graduated line with 0 on the left side as “no pain” and 10 on the right side as “the worst pain.” The physicians rated specific pain scores according to the positions marked by patients on the line.

Quality of life is as follows. The living quality after treatment was assessed by the 36-item short form (SF-36) health survey [11], which consisted of eight parts and was scored out of 100, with a higher total score indicating a better quality of life.

### 2.5. Statistical Disposal

In this work, GraphPad Prism 7 and SPSS 26.0 were used to process the data (GraphPad Software, San Diego, USA) for picture drawing. Count data were tested by *X*^2^ test and represented as *n* (%), and measurement data were *t* test and $\overset{¯}{x}\pm s$. The differences were statistically remarkable when *P* < 0.05.

## 3. Results

### 3.1. Comparison of Clinical Indexes

The clinical indexes in the treatment group after treatment were remarkably better than those in the control group (*P* < 0.05), as detailed in Table 2.

### 3.2. Comparison of Clinical Efficacy

The results indicated that the treatment group had a remarkable higher number of cured cases than the control group (*P* < 0.05), with no remarkable difference in the numbers of improved and ineffective cases of both groups (*P* > 0.05), which was detailed in Table 3.

### 3.3. Comparison of Mobility of Fingers

After treatment, the mean TAM in the treatment group was remarkably higher than that in the control group (*P* < 0.001), which was detailed in Figure 1.

### 3.4. Comparison of Pain Relief

The VAS score after treatment in the treatment group was remarkably lower than that in the control group (*P* < 0.001), which was detailed in Figure 2.

### 3.5. Comparison of Quality of Life

After treatment, the mean SF-36 score in the treatment group was remarkably higher than that in the control group (*P* < 0.001), as detailed in Figure 3.

## 4. Discussion

CTS is a common peripheral nerve entrapment disease in clinic [12], whose pathological manifestations are chronic inflammatory edema and thickening of transverse carpal ligament, compression and degeneration of median nerve, and adhesion of the peripheral tissues [13]. The median nerve, which is composed of the anterior rami of the spinal nerve C_6_-T_1_, descends between the flexor digitorum superficialis and flexor digitorum profundus into the wrist and crosses the carpal tunnel to reach the palm of the hand on the deep side, distributing over the partial skin of the palm and dorsal parts of the index, middle, and the ring fingers [14, 15]. CTS mostly occurs in manual workers, but with the popularization of computers in recent years, its incidence has increased dramatically.

Pain and numbness are the most frequent clinical symptoms in patients with CTS [16] whose current treatments are mainly conservative therapies that are ineffective and time-consuming and the appropriate treatments remain unclear. Some scholars [17] believe that when the median nerve is compressed, the nerve blood circulation will be affected, resulting in ischemic edema and congestion, leading to nutritional impairment and subsequent nerve atrophy which induces the development of CTS. CTS belongs to the category of flaccidity syndrome and tendon injury in traditional Chinese medicine. *Suwen-Yinyang Yingxiang Dalun (The Great Treatise on Yin and Yang's reflection of signs)* says that “blockage of qi brings about pains, injury of form leads to swelling.” CTS is mostly caused by the lack of healthy energy in the body and weiqi's insecurity of defense, which induces the invasion of wind pathogen [18]. Acupuncture and moxibustion at acupoints can dredge the meridians and collaterals and induce diuresis to alleviate edema and pain, thereby reducing the volume of carpal tunnel contents and alleviating the compression of median nerve. Animal experiments have also fully confirmed [19] that the stimulation of acupuncture and moxibustion can promote the regeneration of peripheral nerves. In addition, acupotomy can release the nerve compression with remarkable efficacy while avoiding incisions on patients. It provides the possibility of recovery of the median nerve by loosening the transverse carpal ligament, releasing the pressure on the carpal tunnel and the nerve compression, which serves to alleviate muscle tension and reduce wrist pain, as confirmed in a study by Chen et al. [20].

The study was conducted using a randomized controlled trial, drawing on previous treatment experience. Patients in the control group was treated with hot compress, oral medication, and local injection during hospitalization, while the treatment group received acupotomy and electroacupuncture therapy on top of the above treatments. In terms of clinical effects, the treatment group after treatment had a remarkably higher cure rate than the control group (*P* < 0.05), probably because acupotomy reduced the compression on median nerve in the carpal tunnel by cutting and loosening the transverse carpal ligament, addressing the cause of the disease at its source [21]. Some scholars believe that [22, 23] the acupotomy treatment of CTS improves blood circulation, accelerates metabolism, and better repairs muscle ligament injury. Electroacupuncture promotes the repair of median nerve and the recovery of wrist function and can also dredge local meridian qi [24]. In contrast, although the treatment plan of hot compress, oral medication, and local injection can reduce the clinical symptoms to a certain extent, the sustained efficacy is short and the disease are easy to relapse [25]. In terms of pain alleviation and finger mobility, the treatment group did better than the control group, indicating that acupotomy combined with electroacupuncture therapy can promote the finger mobility and relieve the pain efficaciously, so as to achieve the purpose of treating peripheral nerve injuries and restoring their function.

In conclusion, acupotomy combined with electroacupuncture therapy has a high clinical application value in the treatment of CTS. This combination can increase finger mobility, reduce discomfort, and enhance quality of life. Further research will support the development of a better regimen. Limited by the research conditions, the study has a small sample size and a short follow-up course, of which the expansion is required to further validate the effectiveness of study in the future.

## Figures and Tables

**Figure 1:** Comparison of mobility of fingers after treatment (mean ± SD). Notes: the transverse axis was the treatment group and the control group, and the longitudinal axis was the TAM (degrees). The mean TAM in the treatment group and the control group was 181.03 ± 14.22 degrees and 135.33 ± 12.92 degrees, respectively. ∗ suggested remarkable differences in terms of the mean TAM between both groups (*t* = 13.028, *P* < 0.001).

**Figure 2:** Comparison of pain relief (mean ± SD). Notes: the transverse axis was the treatment group and the control group, and the longitudinal axis was the VAS score (points). The VAS scores in the treatment group and the control group were 2.90 ± 1.27 points and 4.27 ± 1.14 points, respectively. ∗ suggested remarkable differences in terms of VAS scores between both groups (*t* = 4.397, *P* < 0.001).

**Figure 3:** Comparison of SF-36 score (mean ± SD). Notes: the transverse axis was the treatment group and the control group, and the longitudinal axis was the SF-36 score (points). The mean SF-36 scores in the treatment group and the control group were 66.47 ± 4.51 points and 57.77 ± 4.84 points, respectively. ∗ suggested remarkable differences in terms of the mean SF-36 scores between both groups after treatment (*t* = 7.203, *P* < 0.001).

**Table 1:** Comparison of clinical data.

Items	Treatment group (*n* = 30)	Control group (*n* = 30)	*X* ^2^/*t*	*P*
Gender			0.278	0.598
Male/female	13/17	11/19		
Mean age (mean ± SD, years)	44.90 ± 15.88	45.90 ± 15.99	0.243	0.809
BMI (mean ± SD, kg/m^2^)	19.87 ± 0.92	20.14 ± 0.84	1.187	0.240
Course of disease (mean ± SD, months)	2.10 ± 0.88	1.93 ± 0.83	0.770	0.445
Previous treatments				
Wrist immobilization brace	20 (66.67)	21 (70.00)	0.077	0.781
Therapeutic ultrasound	3 (10.00)	4 (13.33)	0.162	0.688
Topical corticosteroid injection	5 (16.67)	2 (6.67)	1.241	0.265
Low-level laser therapy	2 (6.67)	3 (7.14)	0.218	0.640
Education levels				
Junior college and above	6 (20.00)	4 (13.33)	0.480	0.488
High school	4 (13.33)	3 (10.00)	0.162	0.688
Middle school	11 (36.67)	14 (33.33)	0.617	0.432
Primary school	6 (20.00)	4 (13.33)	0.480	0.488
Illiteracy	3 (10.00)	5 (16.67)	0.577	0.448
Residence (*n* (%))			0.067	0.795
Urban area	14 (46.67)	13 (43.33)		
Rural area	16 (53.33)	17 (56.67)		

**Table 2:** Comparison of clinical indexes (mean ± SD).

Groups	*n*	Time from treatment to pain relief (d)	Time of numbness relief (d)	Distension sensation scores (points)
Treatment group	30	5.97 ± 1.450	5.90 ± 2.01	1.10 ± 0.92
Control group	30	9.50 ± 1.590	7.30 ± 1.86	2.03 ± 0.72
*t*		8.985	2.800	4.360
*P*		<0.001	<0.050	<0.050

**Table 3:** Comparison of clinical efficacy (*n* (%)).

Groups	*n*	Cured	Improved	Ineffective
Treatment group	30	17 (56.67)	11 (36.67)	2 (6.67)
Control group	30	9 (30.00)	14 (46.67)	7 (23.33)
*X* ^2^		4.344	0.617	3.268
*P*		<0.050	0.432	0.071

## Data Availability

Data to support the findings of this study is available on reasonable request from the corresponding author.
